This article has been retracted.

# Insomnia, sleepiness, anxiety and depression among different types of gamers in African countries

**DOI:** 10.1038/s41598-020-58462-0

**Published:** 2020-02-06

**Authors:** F. A. Etindele Sosso, D. J. Kuss, C. Vandelanotte, J. L. Jasso-Medrano, M. E. Husain, G. Curcio, D. Papadopoulos, A. Aseem, P. Bhati, F. Lopez-Rosales, J. Ramon Becerra, G. D’Aurizio, H. Mansouri, T. Khoury, M. Campbell, A. J. Toth

**Affiliations:** 1 Center for Advanced Studies in Sleep Medicine, Hopital du Sacré-Coeur de Montreal, Research Center of Cognitive Neurosciences, Institut Santé et Société, Université du Québec à Montreal, Québec, Canada; 2 School of Social Sciences, Department of Psychology, International Gaming Research Unit and the Cyberpsychology Group, Nottingham Trent University, Nottingham, UK; 3 School of Health, Medical and Applied Sciences, Physical Activity Research Group, Central Queensland University, Rockhampton, Australia; 4 Center for Research in Nutrition and Public Health, Autonomous University of Nuevo Leon, Monterrey, N.L. Mexico; 5 Centre for Physiotherapy and Rehabilitation Sciences, Jamia Millia Islamia, New Delhi, India; 6 Department of Biotechnological and Applied Clinical Sciences, University of L’Aquila, L’Aquila, Italy; 7 Department of Pulmonology, Army Share Fund Hospital, Athens, Greece; 8 Faculty of Medicine, Université de Montréal, Montréal, Québec, Canada; 9 Department of Biomedical sciences, Faculty of Arts and Sciences, University of Montréal, Montréal, Québec, Canada; 10 Department of Physical Education and Sport Sciences, University of Limerick, Limerick, Ireland; 11 Innovation and Evaluation in Health Psychology, Faculty of Psychology, Autonomous University of Nuevo Leon, Monterrey, Nuevo Leon, Mexico; 12 Lero Irish Software Research Centre, University of Limerick, Limerick, Ireland

**Keywords:** Sleep, Addiction, Anxiety, Depression, Human behaviour

## Abstract

Gaming has increasingly become a part of life in Africa. Currently, no data on gaming disorders or their association with mental disorders exist for African countries. This study for the first time investigated (1) the prevalence of insomnia, excessive daytime sleepiness, anxiety and depression among African gamers, (2) the association between these conditions and gamer types (i.e., non-problematic, engaged, problematic and addicted) and (3) the predictive power of socioeconomic markers (education, age, income, marital status, employment status) on these conditions. 10,566 people from 2 low- (Rwanda, Gabon), 6 lower-middle (Cameroon, Nigeria, Morocco, Tunisia, Senegal, Ivory Coast) and 1 upper-middle income countries (South Africa) completed online questionnaires containing validated measures on insomnia, sleepiness, anxiety, depression and gaming addiction. Results showed our sample of gamers (24 ± 2.8 yrs; 88.64% Male), 30% were addicted, 30% were problematic, 8% were engaged and 32% were non-problematic. Gaming significantly contributed to 86.9% of the variance in insomnia, 82.7% of the variance in daytime sleepiness and 82.3% of the variance in anxiety [p < 0.001]. This study establishes the prevalence of gaming, mood and sleep disorders, in a large African sample. Our results corroborate previous studies, reporting problematic and addicted gamers show poorer health outcomes compared with non-problematic gamers.

## Introduction

With the popularity of consoles, such as the PlayStation and the X-box, and the possibility to use various applications on smartphones and tablets due to easy access to Wi-Fi and mobile data, gaming has become a part of life in Africa, similarly to Europe and North America. Recently, some reports estimated that African countries such as Nigeria have over 146,866,356 active mobile phone lines, with mobile users interested in available online entertainment content (BBC 2016), which may negatively impact on users’ health in some cases^1,2^. It was also suggested by Wittek *et al*.^3^, when assessing prevalence rates and predictors of video game addiction in a multicultural sample including native Norwegians and immigrants, that the geographical region where an individual is born may play an important role in addictive behavior. They reported there were more addicted gamers who originated from African, Asian and central American countries compared with gamers born in Europe and North America. Prevalence of gaming disorders was reported in Europe, Asia and North America^3–9^; while no data exist for prevalence in African countries as well as their association with sleep and mood disorders.

New technologies, including internet use and gaming, influence lifestyle behaviours, which, may affect mental health and lead to the development of addictive behaviors, particularly in young individuals^9–12^. Gaming disorder is now included under the addictive behaviors category in the 11^th^ update of the World Health Organization’s International Classification of Diseases (ICD-11). *Gaming Disorder* generally refers to a diagnosis characterized by uncontrollable and persistent playing of video and digital games that is harmful to an individual’s wellbeing, often leading to addictive behaviors. Rather than engaging in the offline world, an addicted user devotes the majority of his or her time to gaming. The addicted gamer often isolates him/herself from others, ignores more important responsibilities, and is often preoccupied with obtaining higher status/rankings/achievements in his/her favorite computer game. This may be the case for using gambling and gaming on computers and consoles as the available evidence indicates gaming with wireless devices, such as smartphones, does not appear to be problematic^13^. Similar evidence was reported for the use of online social networking sites and Massively Multiplayer Online games (MMOs)^11,14^.

Although research in the area of Gaming Disorder is progressing^15^, few studies have explored the association between gaming behavior and sleep disorders^16–25^. Although some sleep disorders are consequences of cortical imbalances^26^, including insomnia and restless leg syndrome, lifestyle behaviours can also influence their incidence considerably^27–30^. Sleep disorders increase when individuals have mood and anxiety disorders, deficits in attention or perception, or when individuals live under stressful conditions (i.e., low income, and working night shifts)^31–35^. On the other hand, anxiety and depression are often associated with occurrence of sleep disturbances in many studies; showing an interplay between these three neuropsychiatric diseases sharing several neurotransmitters like serotonin and dopamine (both involved in sleep, cognition, emotion and behaviour)^36–38^. Behavioural and medical risk factors (i.e., high-blood pressure, obesity, smoking)^39–41^, lower quality of life and a stressful environment have all been associated with the occurrence of sleep disorders^27^. Sleep disorders affect the normal functioning of an individual by decreasing vigilance, attention, performance at work and increasing cognitive impairments^42,43^. Prevalence and incidence of sleep disorders, anxiety and depression are poorly documented in Africa, which creates a gap in the sleep medicine field^44,45^.

The use of smartphones, computers, consoles, and online video games can disturb the circadian process^46–50^. It has been reported that the presence of or exposure to light can disturb the circadian rhythm, the melatonin cycle and cerebral plasticity, which may affect the quality and duration of sleep^26,51^. To fall asleep, neuronal inhibition increases, while cortical excitation decreases. During this process, different sleep stages occur, and neurons build new networks while consolidating memory. Wireless devices including smartphones, laptops or tablets may therefore affect sleeping patterns as they rely on backlighting. Recent reports suggest a higher incidence and prevalence of behavioral disturbances in children and adolescents exposed to screen-based technologies such as computer, tablets and smartphone; and playing online games for several hours a week at home^6,10,52^. Considering the impact of light, a stressful environment and visual stimulation on sleep mechanisms and the risk excessive gaming may pose for sleep and psychopathology, it may be hypothesised that gaming decreases sleep quality and increases sleep disorders and psychopathological symptoms. As of yet, this hypothesis has not been reported in the available scientific literature. Some associations or indirect links have been found between the use of technologies (the internet, video games, and electronic media) and factors associated with sleep (sleep quality, sleep duration, and sleep habits) for preadolescents, adolescents and older adults^16–25^, but a clear association between gaming and sleep disorders has not yet been established.

There is a gap in knowledge regarding the assessment of gaming behaviors and their impact on sleep in developing and low- and middle-income countries. There is a lack of data particularly for African countries, which face the same problems in comparisons to other countries related to the use of the internet and gaming^1,2,53–55^. Given the lack of knowledge in the fields of gaming, mood disorders and sleep disorders in African countries, the purpose of this study is to investigate (1) the prevalence of insomnia, excessive daytime sleepiness, anxiety and depression among African gamers, (2) the association between these four conditions and different types of gamers (non problematic, engaged, problematic and addicted) and (3) assess the predictive power of socioeconomic markers (education, age, income, marital status and employment status) on insomnia, excessive daytime sleepiness, anxiety and depression of gamers.

## Methods

### Ethics committee

This is a secondary analysis of data collected during the project MHPE approved by the Faculty of Arts and Science of the University of Montreal (CERAS-2015-16-194-D) and by the administrator or dean of the universities at which recruitment took place, in accordance with the declaration of Helsinki. All participants were recruited through the respective admissions offices and provided their informed consent prior to volunteering in the study. All participants were contacted via the email lists of the admission office or by an individual inside each participating institution. The data were secured outside the public network in an external server and were shared only with the main investigators involved in the project.

### Data collection

The study was conducted in 2 low- (Rwanda, Gabon), 6 lower-middle (Cameroon, Nigeria, Morocco, Tunisia, Senegal, Ivory Coast) and 1 upper-middle income countries (South Africa). The nine countries chosen in this study were included because (1) their citizens have greater access to gaming devices, (2) they have been ranked in the top 20 of highly developed African countries in terms of technology use, internet connectivity and potential for the market of gaming and gambling (i.e., measured via the increased number of gamers, presence of casinos, and expenses for gaming purposes) in the last four years, according to the most recent annual report of the International Telecommunication Union (ITU 2017), who regularly publish “measuring the information society report”, which is the world’s reference in terms of data related to the development of communications, technologies and connectivity^56^.

The participants who formed this convenience sample were contacted by email. The online questionnaire included a consent form on the second page, following a description of the study in French and English. Consent was required to participate in this project. The average time to answer all questions was 20 minutes. The questionnaire could only be completed once by participants with the same email address, and duplicates and incomplete forms were removed. Responses were collected between November 2015 and June 2017.

### Measures

#### Insomnia severity index (ISI)

This questionnaire is widely used to assess insomnia and associated parameters, including lack of sleep and sleep quality. It was developed by Morin *et al*. in 2001^57,58^. The internal consistency of the ISI was excellent (Cronbach’s α = 0.92), and each individual item showed adequate discriminative capacity (*r = *0.65–0.84). The area under the receiver operator characteristic curve was 0.87 and suggested that a cut-off score of 14 was optimal (82.4% sensitivity, 82.1% specificity, and 82.2% agreement) for detecting clinical insomnia. An ISI score between 0 and 7 is insomnia which is considered clinically non-significant, between 8 and 14 as subthreshold insomnia, between 15 and 21 as a moderate clinical insomnia, and between 22 and 28 indicates severe clinical insomnia^57,58^.

#### Epworth sleepiness scale (ESS)

The Epworth Sleepiness Scale is a simple and reliable instrument that has been used worldwide (Johns, 1991). This test assesses drowsiness levels throughout the day, also known as excessive daytime sleepiness. This test also indicates if a certain degree of drowsiness may warrant a visit to the doctor and a more thorough assessment to diagnose a sleep respiratory disorder. The test consists of eight questions (0 to 3 points) and is completed in less than five minutes. If the participant scores 9 points or fewer, it is considered normal. If the participant scores 10 points or more, an appointment should be made with a sleep specialist. The Epworth scale only quantifies subjective drowsiness (interpreted by the participant) regardless of its association with a sleep disorder.

#### The hospital anxiety and depression scale (HADS)

This is a self-administered scale including 14 items, divided into two subscales of seven items (Anxiety or HADS-A, Depression or HADS-D). It contains no somatic items that can be confused with the symptomatic manifestations of a disease. Each item is scored on a scale of 0 to 3. A score is generated for each of the two sub-scales and for the entire HADS (HADS-T). The scoring is similar for anxiety and depression and there are three categories of symptomatic levels: non-cases or asymptomatic ones (scores ≤ 7); probable or borderline cases (scores 8–10); clearly or clinically symptomatic cases (scores ≥ 11). The duration of administration is approximately five minutes and psychometric properties are detailed in previous studies^59,60^.

#### The game addiction scale short form (GAS-SF)

Initially developed by Lemmens *et al*. in 2009 with 21 items and a Cronbach’s α of 0.82 to 0.87^61^, the 7-item GAS-SF was validated later and is considered an adequate tool for assessing problematic online gaming with whatever device is used for gaming purposes according to recent studies^62,63^. GAS-SF allows the following classifications: addicted gamers (scoring three or more on four core items [relapse, withdrawal, conflict and problems]), problem gamers (scoring three or more on two or three of the four same items), engaged gamers (scoring three or more on the first three items [salience, tolerance, and mood modification], but who do not score three or above on the other items), and normal gamers or non-problematic gamers (gamers not classified as addicted, problem, or engaged)^64,65^.

#### The gaming period

It was measured in terms of the time spent gaming per week for each participant with one-item “how many hours are you gaming per week?”. Based on responses, an average time of gaming per month was computed for all the participants of each country.

The demographics which were collected are the following: age, sex (i.e., man or woman), income [the global family income (parent’s household & income if they were only student) and the personal income (if they were workers or student-workers) both categorized as low, middle and high], education (categorized as primary, high school, bachelor, master, doctorate, or post-doctorate), marital status [classified as single, married, or engaged (for people in relationships without marriage)] and employment status (classified as only student, student and employed, or employed).

### Statistical analysis

The normal distribution of the data was analyzed using a Shapiro Wilk test. Unpaired sample t-tests were used to compare difference in insomnia, sleepiness, anxiety and depression for males vs. females. A one-way ANOVA with a Bonferroni multiple-comparison post-hoc correction was performed to analyze differences between the four types of gamers and their level of anxiety, depression, insomnia and excessive daytime sleepiness. Then, 4 multiple linear regression analyses were performed (with normal gaming as reference category) to compare the odds for having these conditions (which are dependent variables) for different levels of gaming. The independent variables “months of being a gamer” and “number of hours of gaming per week” were coded as continuous variables. “Employment status”, “sex”, “marital status”, “income”, “education” and “gender” were coded as categorical variables. The dependent variables “insomnia”, “excessive daytime sleepiness”, “anxiety” and “depression” were coded as continuous variables. Preliminary analyses were performed to verify the respect of the assumptions of normality, linearity, multicollinearity and homoscedasticity. All the statistical tests used an alpha of 0.05 as level of significance. Data analysis was performed using PRISM (Graph Pad Prism, version 7.0.0.159, Graph pad software) and SPSS version 25 (IBM Corp, Armonk, NY, USA).

## Results

The Characteristics of the sample are detailed in Table 1. A total of 53,634 invitations were sent to potential participants and 12,680 forms were returned (response rate = 23.64%). After removing incomplete forms (n = 2,114), the final sample included 10,566 gamers (3381 non problematic gamers, 845 engaged gamers, 3170 problematic gamers and 3170 addicted gamers). Participants were university students aged between 18 and 40 years old (24 ± 2.8 years). In this population of gamers, the majority of participants were aged between 18 and 24 years (6258 men and 876 women). Women represented 11.36% of the participants. Most of the respondents (98.77%) were undergraduates (9247 men and 1189 women). The majority of participants (66.02%) reported a middle income (6251 men and 724 women) and 3036 (28.73%) reported a high income; while a larger proportion of women reported a low income (35.5%, n = 426) compared with men (1.38%, n = 129). Also, more than 94% of the participants were single (9278 men and 1129 women). Finally, 72.08% of the participants did not work while studying (n = 7616), while 24.07% of them reported working alongside their studies (n = 2543) and the rest were only employees (n = 407).

**Table 1:** Sociodemographic characteristics of participants where age, education, income, marital status, employment status and different types of gamers are reported for the entire sample.

Sociodemographic variables	Total sample (N = 10566, 100%)	Men (n = 9366, %)	Women (n = 1200, %)	Non-problematic Gamers (n = 3381, %)	Engaged Gamers (n = 845, %)	Problematic Gamers (n = 3170, %)	Addicted Gamers (n = 3170, %)
**Age (years)**							
*18–24*	7134 (67.52%)	6258 (66.82%)	876 (73%)	2643 (78.17%)	753 (89.11%)	3089 (97.44%)	649 (20.47%)
*24–30*	3168 (29.98%)	2871 (30.65%)	297 (24.75%)	704 (20.82%)	75 (8.87%)	79 (2.5%)	2310 (72.87%)
*30–36*	257 (2.43%)	230 (2.46%)	27 (2.25%)	30 (0.88%)	15 (1.78%)	2 (0.06%)	210 (6.63%)
*36–42*	7 (0.07%)	7 (0.07%)	0	4 (0.12%)	2 (0.24%)	0	1 (0.03%)
*42–48*	0	0	0	0	0	0	0
**Education (degree)**							
*Bachelor*	10436 (98.77%)	9247 (98.73%)	1189 (99.08%)	3293 (94.44%)	810 (95.86%)	3167 (99.9%)	3166 (99.87%)
*Master*	128 (1.21%)	117 (1.25%)	11 (0.92%)	88 (5.56%)	33 (3.90%)	3 (0.1%)	4 (0.13%)
*Doctorate*	2 (0.02%)	2 (0.02%)	0	0	2 (0.24%)	0	0
*Postdoctorate*	0	0	0	0	0	0	0
**Income**							
*Low*	555 (5.25%)	129 (1.38%)	426 (35.5%)	500 (14.79%)	46 (5.44%)	9 (0.28%)	0
*Middle*	6975 (66.02%)	6251 (66.74%)	724 (60.33%)	2857 (84.5%)	697 (73.76%)	3027 (95.49%)	394 (12.43%)
*High*	3036 (28.73%)	2986 (31.88%)	50 (4.17%)	24 (0.71%)	102 (20.8%)	134 (4.23%)	2776 (87.57%)
**Marital status**							
*Single*	10407 (98.5%)	9278 (99.06%)	1129 (94.08%)	3359 (99.35%)	820 (97.04%)	3156 (99.56%)	3072 (96.9%)
*Engaged*	155 (1.47%)	85 (0.9%)	70 (5.83%)	18 (0.53%)	25 (2.96%)	14 (0.44%)	98 (3.09%)
*Married*	4 (0.03%)	3 (0.04%)	1 (0.09%)	4 (0.12%)	0	0	0
**Employment status**							
*Student only*	7616 (72.08%)	6524 (69.66%)	1092 (91%)	3209 (94.91%)	786 (93.02%)	2792 (88.08%)	829 (26.15%)
*Employed*	407 (3.85%)	305 (3.26%)	102 (8.5%)	53 (1.57%)	59 (6.98%)	78 (2.46%)	217 (6.85%)
*Student & employed*	2543 (24.07%)	2537 (27.08%)	6 (0.5%)	119 (3.52%)	0	300 (9.46%)	2124 (67%)

Table 2 indicates that the favourite gaming device was the smartphone, followed by computers and consoles. Tablets were the device least used for gaming. This finding was similar for all countries except for Gabon, where participants reported using their tablets more than smartphones and consoles. The largest number of smartphone gamers were found in South Africa (58.14%), followed by Morocco (51.9%) and Cameroon (48.08%). South Africa also had the largest number of computer gamers (31%) followed by Morocco (37.62%) and Nigeria (46.61%). Cameroon had the largest proportion of gamers using consoles (27.95%), followed by Rwanda (21.4%) and South Africa (7.22%). Gabon was the country with the largest proportion of gamers using tablets (48.33%), followed by South Africa (3.64%) and Nigeria (6.4%). Table 2 also shows that the majority of participants across all countries were categorized as non-problematic gamers (n = 850 (32.95%) for South Africa, n = 480 (32.97%) for Cameroon, n = 350 (38.54%) for Ivory Coast, n = 146 (32.52%) for Gabon, n = 673 (36.76%) for Morocco, n = 472 (36.37%) for Nigeria, n = 261 (29.09%) for Rwanda, n = 261 (30.85%) for Senegal and n = 88 (29.23%) for Tunisia. In Tunisia, participants were found to spend the highest average time gaming per week (20 h ± 2.5 hours), followed by Morocco (18 ± 2.5 hours) and South Africa (17 ± 2.5 hours). In Gabon and Senegal participants played fewer hours per week (respectively 6 ± 0.5 hours and 6 ± 2.5). In Tunisia, participants reported the longest period where they considered themselves as gamers (26 ± 2 months), followed by Morocco (18 ± 2 months) and Cameroon (19 ± 1 months). In Rwanda participants reported the lowest average gaming period, i.e., 10 ± 2 months.

**Table 2:** Descriptive epidemiology of gaming among the nine African countries where prevalence of gaming, mean hours of gaming per week, period from when participant considered himself a gamer and type of device used for gaming purposes are described with age and sex.

Country	Total	Age	Men	Women	Mean Hours of Gaming/week	Mean Months of Gaming/gamer	Addicted Gamers	Problematic gamers	Engaged Gamers	Non problematic Gamers	Gamers using smartphones	Gamers using tablets	Gamers using computers	Gamers using consoles
**South Africa**	2580	21 ± 3	2194 (85.04%)	386 (14.96%)	17 ± 2.5	14 ± 2	820 (31.78%)	805 (31.2%)	105 (4.07%)	850 (32.95%)	1500 (58.14%)	94 (3.64%)	800 (31%)	186 (7.22%)
**Cameroon**	1456	19 ± 3	1300 (89.28%)	156 (10.72%)	10 ± 1.75	19 ± 1	456 (31.32%)	435 (29.87%)	85 (5.84%)	480 (32.97%)	700 (48.08%)	63 (4.33%)	286 (19.64%)	407 (27.95%)
**Ivory Coast**	908	23 ± 2	785 (86.45%)	123 (13.55%)	12 ± 1.25	13 ± 1	278 (30.62%)	227 (25%)	53 (5.84%)	350 (38.54%)	230 (25.33%)	58 (6.39%)	520 (57.27%)	100 (11.01%)
**Gabon**	449	20 ± 2	414 (92.2%)	35 (7.8%)	6 ± 0.5	15 ± 1	134 (29.84%)	123 (27.4%)	46 (10.24%)	146 (32.52%)	153 (34.08%)	217 (48.33%)	62 (13.8%)	17 (3.79%)
**Morocco**	1831	20 ± 2	1662 90.77%)	169 (9.23%)	18 ± 2.5	18 ± 2	504 (27.53%)	497 (27.14%)	157 (8.57%)	673 (36.76%)	950 (51.9%)	41 (2.24%)	689 (37.62%)	151 (8.24%)
**Nigeria**	1298	25 ± 2	1147 (88.37%)	151 (11.63%)	12 ± 2.25	13 ± 1.75	350 (26.96%)	350 (26.96%)	126 (9.71%)	472 (36.37%)	456 (35.13%)	83 (6.4%)	605 (46.61%)	154 (11.86%)
**Rwanda**	897	25 ± 1	809 (90.19%)	88 (9.81%)	8 ± 2	10 ± 2	260 (29%)	230 (25.64%)	146 (16.27%)	261 (29.09%)	371 (41.36%)	18 (2.01%)	316 (35.23%)	192 (21.4%)
**Sénégal**	846	22 ± 2	770 (91%)	76 (9%)	6 ± 2.5	11 ± 0.25	211 (24.94%)	320 (37.83%)	54 (6.38%)	261 (30.85%)	387 (45.74%)	7 (0.83%)	366 (43.26%)	86 (10.17%)
**Tunisia**	301	26 ± 4	285 (94.68%)	16 (5.32%)	20 ± 2.5	26 ± 2	57 (18.94%)	83 (27.58%)	73 (24.25%)	88 (29.23%)	100 (33.22%)	26 (8.64%)	94 (31.23%)	81 (26.91%)

Figure 1 shows the distribution of the four conditions among our population of gamers. Being a non-problematic gamer (NG) or an engaged gamer (EG) is associated with the lowest mean score of insomnia (respectively 6 ± 1.2 and 6.2 ± 1), excessive daytime sleepiness (respectively 5 ± 0.5 and 6 ± 0.5), anxiety (respectively 4 ± 0.6 and 4.7 ± 0.7) and depression (respectively 4 ± 0.4 and 4.5 ± 0.7), with a small increase for each when NG are compared with EG. However, these conditions are more prevalent for problematic gamers (PG) and addicted gamers (AG) with respectively 14 ± 1 and 18 ± 1 for insomnia, 11 ± 0.5 and 14 ± 0.75 for excessive daytime sleepiness, and 9 ± 1 and 11.5 ± 0.5 for anxiety. The findings show significant differences across the groups for insomnia, excessive daytime sleepiness and anxiety, with more problematic gaming increasingly associated with higher scores on daytime sleepiness and anxiety. The results also reveal that none of the gaming categories in the present paper were associated with depression; even if PG and AG still have higher mean scores than NG and EG (Fig. 1D).

**Figure 1:** Comparison and differences of neuropsychiatric diseases between the categories of gamers. A one-way ANOVA with a Bonferroni multiple-comparison post-hoc correction was performed to analyze differences between normal/non problematic gamers (NG) vs. engaged gamers (EG) vs. problematic gamers (PG) vs. addicted gamers (AG). (**A**) Severity of insomnia (measured with ISI) for NG, EG, PG and AG. (**B**) Symptoms of excessive daytime sleepiness (measured with the ESS) for NG, EG, PG and AG. (**C**) Severity of anxiety symptoms (measured with HADS-A) for NG, EG, PG and AG. (**D**) Severity of depression symptoms (measured with HADS-B) for NG, EG, PG and AG. *p < 0.05. **p < 0.01. ***p < 0.001. All the statistical tests used an alpha of 0.05 as level of significance.

Table 3 shows the results of the multiple regression analyses where age, sex, income, marital status, education, employment status and type of gaming (with non-problematic gaming as a reference category) were regressed upon the neuropsychiatric conditions. In Model 1 which predicts insomnia, the independent variables problematic gamers (β = 0.72), addicted gamers (β = 1.8), man (β = 0.347), age [β (24–30) = 0.752)], education [β (postdoctorate) = 0.08], high income (β = 0.347) and marital status [β (engaged) = 0.23] were positively associated with insomnia. The independent variables age [β (30–36) = −0.09; β (36–42) = −0.148)], being married (β = −0.483) and being a student and employed (β = −0.263) were negatively associated with insomnia. All these independent variables significantly contributed to 89% of the variance [F (25, 10541) = 257.71, p < 0.001] in insomnia. Model 2 predicted excessive daytime sleepiness. The independent variables problematic gamers (β = 0.189), addicted gamers (β = 387), age [β (24–30) = 0.218)] and high income (β = 0.157) were positively associated with excessive daytime sleepiness. The independent variables age [β (30–36) = −0.049; β (36–42) = −0.848)], being postdoctorate (β = −0.248), marital status [β (engaged) = −0.246; β (married) = −0.272] and employment status [β (worker) = −0.048; β (student-worker) = −0.263] were negatively associated with excessive daytime sleepiness. Together, these variables explained 84% of the variance [F (25, 10541) = 175.86, p < 0.001] in daytime sleepiness. Model 3 predicted anxiety. The independent variables problematic gamers (β = 0.238), addicted gamers (β = 0.574), sex [women (β = 0.09)], age [β (24–30) = 0.294); β (42–48) = 0.192], income [β (middle) = 0.168] and being a student-worker (β = 0.216) were positively associated with anxiety. Negative associations with anxiety were found with marital status [β (engaged) = −0.243; β (married) = −0.291]. All these predictors significantly contributed to explaining 83% of the variance in anxiety scores [F (25, 10541) = 212.96, p < 0.001]. Finally, model 4 predicted depression [variance of 76%, F (25, 10541) = 214.48, p < 0.001] by problematic gamers (β = 0.231), addicted gamers (β = 0.348), sex [women (β = 0.073)], age [β (36–42) = 0.112; β (42–48) = 0.1)] and being student-worker (β = 0.185).

**Table 3:** Results of the Multiple Regression Analyses where age, sex, income, marital status, education, employment status and type of gaming [with non-problematic gaming, sex (male), age (18–24), education (bachelor), income (low), marital status (single) and employment status (student only) used as reference categories for each variables) were regressed upon the neuropsychiatric diseases. Model 1: multiple linear analysis with insomnia as dependent variable. Model 2: multiple linear analysis with excessive daytime sleepiness as dependent variable. Model 3: multiple linear analysis with anxiety as dependent variable. Model 4: multiple linear analyses with depression as dependent variable. B = unstandardized regression coefficient. β = standardized regression coefficient. SE = standard error. t = t-test statistic. Sig. = Significance level (p-value), *p < 0.05. **p < 0.01. ***p < 0.001. ΔR^2^ = change in variance. F = statistic of Fisher.

Model 1: Prediction of Insomnia									
Model summary						95% Confidence Interval		Precision of prediction	
Variables	B	SE	β	t	Sig.	Lower Bound	Upper Bound	ΔR^2^	F
**Type of Gamers**								0.89	(25, 10541) = 251.87, p <0.001
Engaged	0.861	0.002	0.23	9.748	0.523	−0.21	2.458		
Problematic	5.984	1.007	0.72	53.416	0.000***	0.798	3.862		
Addicted	10.608	3.086	1.8	70.975	0.000***	1.153	4.936		
**Sex**									
Female	0.842	0.26	0.09	12.406	0.692	−0.263	2.074		
**Age**									
24–30	2.785	1.005	0.752	29.741	0.000***	0.876	3.429		
30–36	−0.807	0.48	−0.09	−10.118	0.000***	0.785	3.478		
36–42	−1.487	1.044	−0.148	−14.769	0.023*	0.805	4.789		
42–48	1.472	0.945	0.153	12.337	0.92	0.189	1.967		
**Education (degree)**									
Master	0.062	0.041	0.005	6.314	0.741	0.231	2.486		
Doctorate	0.201	0.06	0.002	2.078	0.433	0.199	2.981		
Postdoctorate	1.178	1.031	0.08	11.723	0.032*	0.742	3.476		
**Income**									
Middle	0.412	0.87	0.04	4.259	0.289	0.179	2.008		
High	2.486	1.11	0.347	24.842	0.000***	0.832	3.796		
**Marital status**									
Engaged	2.442	0.474	0.23	24.547	0.000***	0.745	4.018		
Married	−6.475	1.007	−0.483	−12.145	0.000***	0.915	4.903		
**Employment status**									
Employed	−0.475	1.42	−0.041	−1.347	0.412	0.261	2.978		
Student & employed	−12.91	2.742	−0.263	−11.847	0.000***	0.974	5.949		
**Model 2: Prediction of Excessive Daytime Sleepiness**									
**Type of Gamers**								0.84	(25, 10541) = 184.87, p <0.001
Engaged	0.783	0.072	0.248	7.956	0.087	0.196	1.987		
Problematic	1.874	1.094	0.189	18.016	0.000***	0.922	2.824		
Addicted	4.588	1.796	0.387	30.725	0.000***	1.135	4.328		
**Sex**									
Female	0.719	0.417	0.032	7.194	0.108	0.263	1.792		
**Age**									
24–30	2.105	0.746	0.218	21.075	0.000***	0.967	3.897		
30–36	−0.484	0.543	−0.049	−40.88	0.000***	1.685	5.694		
36–42	−0.845	1.044	−0.848	−8.769	0.000***	0.495	2.897		
42–48	−1.197	0.945	−0.198	−12.649	0.076	−0.189	3.423		
**Education (degree)**									
Master	0.427	0.596	0.043	4.379	0.742	0.171	1.869		
Doctorate	−0.201	0.095	−0.798	−2.706	0.291	0.149	2.001		
Postdoctorate	−1.468	1.207	−0.248	−15.72	0.000***	0.959	2.796		
**Income**									
Middle	1.236	0.478	0.119	12.462	0.642	0.179	1.908		
High	1.487	0.984	0.157	14.985	0.000***	0.872	2.965		
**Marital status**									
Engaged	−2.442	1.706	−0.246	−24.547	0.000***	1.008	3.804		
Married	−2.713	1.007	−0.272	−20.241	0.000***	1.207	3.429		
**Employment status**									
Employed	−0.489	1.42	−0.048	−1.347	0.238	0.324	2.978		
Student & employed	−2.914	2.742	−0.263	−29.85	0.000***	1.004	3.084		
**Model 3: Prediction of Anxiety**									
**Type of Gamers**								0.83	(25, 10541) = 212.96, p <0.001
Engaged	0.964	0.078	0.092	9.269	0.059	0.216	1.872		
Problematic	2.297	1.164	0.238	20.916	0.000***	1.102	2.862		
Addicted	4.895	1.089	0.574	48.804	0.000***	1.078	4.068		
**Sex**									
Female	0.891	0.472	0.09	8.805	0.000***	0.963	2.925		
**Age**									
24–30	2.938	1.005	0.294	29.741	0.000***	1.207	3.764		
30–36	2.307	0.48	0.237	20.358	0.207	−0.285	2.004		
36–42	0.876	0.8	0.184	8.469	0.086	0.308	2.802		
42–48	2.898	1.538	0.192	28.537	0.000***	0.99	3.839		
**Education (degree)**									
Master	0.062	0.041	0.005	6.314	0.742	0.241	1.487		
Doctorate	0.201	0.06	0.0018	2.078	0.291	0.202	2.381		
Postdoctorate	1.178	1.031	0.08	11.723	0.000***	0.769	2.796		
**Income**									
Middle	1.694	1.035	0.168	17.321	0.000***	1.108	3.185		
High	2.194	0.839	0.227	21.842	0.095	0.281	2.062		
**Marital status**									
Engaged	−2.429	1.338	−0.243	−0.243	0.000***	0.946	3.948		
Married	−2.906	0.943	−0.291	−0.291	0.000***	1.078	3.197		
**Employment status**									
Employed	0.275	0.45	0.027	1.347	0.238	0.229	2.978		
Student & employed	2.164	1.5	0.216	20.335	0.000***	0.998	3.907		
**Model 4: Prediction of Depression**									
**Type of Gamers**								0.76	(25, 10541) = 214.48, p <0.001
Engaged	1.789	1.325	0.178	17.906	0.083	0.218	2.108		
Problematic	2.294	1.007	0.231	23.065	0.000***	0.985	3.893		
Addicted	3.476	1.35	0.348	30.196	0.000***	1.203	4.036		
**Sex**									
Female	0.734	0.276	0.073	7.351	0.004**	0.867	2.869		
**Age**									
24–30	1.621	1.603	0.162	16.227	0.073	0.376	2.272		
30–36	0.679	0.125	0.072	6.845	0.176	0.185	2.728		
36–42	1.117	0.698	0.112	11.18	0.045*	0.795	3.787		
42–48	0.987	0.267	0.1	9.922	0.026*	0.708	2.978		
**Education (degree)**									
Master	0.937	0.594	0.092	9.297	0.742	0.197	2.872		
Doctorate	0.489	0.138	0.048	4.902	0.291	0.249	2.488		
Postdoctorate	0.776	0.255	0.077	7.729	0.7	0.742	3.476		
**Income**									
Middle	1.497	1.012	0.148	14.972	0.695	0.209	2.462		
High	1.634	1.106	0.164	16.346	0.678	0.232	2.007		
**Marital status**									
Engaged	−0.972	0.268	−0.092	−9.478	0.000***	1.092	3.178		
Married	−1.798	1.161	−0.176	−17.7	0.000***	1.115	2.903		
**Employment status**									
Employed	1.763	1.045	0.175	17.658	0.238	0.261	2.978		
Student & employed	1.874	1.428	0.185	18.678	0.006**	0.874	5.949		

## Discussion

The aim of this research was to classify the different types of gamers that exist among African university students at universities where gaming devices are readily available and document the presence of insomnia, excessive daytime sleepiness, anxiety and depression in African gamers. Moreover, we aimed to examine associations between these four conditions and the different gamer types (non problematic, engaged, problematic and addicted). Our results corroborate previous studies which reported that problematic gamers and addicted gamers show poorer health outcomes when compared to non-problematic gamers^31,66^.

Our findings are similar with those reported in Asian countries and Europe. Prevalence of gaming disorders in Africans is most closely related to findings in adolescent and student populations in Asian countries, associated with addictive behaviors and a high prevalence of problematic internet use^7^. A number of studies suggests that online gamers with longer weekly gaming hours tend to have more severe depressive and Internet addiction symptoms^67^, as well as sleep disorders^68,69^. In Europe and Asia, problematic gamers also tend to develop somatic and musculoskeletal diseases, due to their poor physical activity and their progressive addiction^7,67,69^. The prevalence is similar for adolescents and students, males and females^9,68,70^. Despite the increase of studies on gaming disorders and technology-related disorders around the world, this topic remains understudied in low-income countries and particularly in Africa. Wittek *et al*. in 2016 showed the differences in prevalence of gaming disorders regarding the place of birth and was among the first to think about the importance of gaming disorders in Africa^3^.

The present study also revealed disparities in the use of gaming devices across different countries in Africa. The most recent annual report of the International Telecommunication Union (ITU 2018) reported that all 9 countries included in this research were ranked among the 20 most developed countries in terms of technologies and connectivity in Africa. Our findings demonstrate that the more developed a country is in terms of connectivity and technologies (i.e., South Africa, Nigeria, Cameroon and Tunisia), the more problematic gamers are found. Regardless of type of gamers and countries in this study, preference was given to smartphone for gaming. This may be due to the price of consoles, which are very expensive relative to salaries common in Africa. The 2017 International Monetary Fund (IMF) annual report demonstrated that the average gross domestic product (i.e., the purchasing power parity per person per year) of included populations remain among the weakest in the world. The average price of a console-based video game, such as the PlayStation 4, is USD300, which equates to nearly a tenth of the annual income of a Cameroonian or a seventh of the annual income of a Rwandan (IMF Annual Report, 2017). This phenomenon can also be explained by how much easier and cheaper it is to purchase a smartphone through an online marketplace (e.g., eBay or Amazon), and then downloading free games using application portals such as the Google Play store or Apple App store. It is easy to download a mobile game on a wireless device and most of these games are free, compared with the expensive price of a DVD game which tends to be priced at an average of USD 40 and often more. This may explain why wireless devices like smartphones and laptops are more popular than classical consoles for gaming in these countries.

The present research found that gaming was associated with sleep disturbances^20,21^. Individually, gaming and using wireless devices are associated with addictive behaviours (i.e., gambling)^10^. Addiction is often associated with mood disorders which are strongly associated with sleep disorders^66,71^. The results of the present study suggest that there is a similar relationship between gaming (specifically online gaming) and the experience of sleep disorders and psychopathological symptoms such as anxiety and depression. Typically, insomnia is more prevalent in elderly populations than in adolescents^72^. However, our findings show that the incidence of insomnia is greater in problematic and addicted compared to non-problematic and engaged adolescent high school and university gamers. However, our results also suggest that the experience of sleep problems may also be influenced by an individuals’ environment, including the respective country individuals reside in, and their social class^66,73,74^. Our findings confirm that there are significant associations between markers of socioeconomic status, such as high income, and insomnia and excessive daytime sleepiness. According to our ANOVAs, the addicted gamers are older, have a higher income and were employed a lot more than the other groups. This is interesting as it suggests a higher income is likely to help individuals sustain a gaming addiction. Moreover, the observation that addicted individuals seem to be older may be attributed to the fact that it takes some time for addiction to develop. Together, these findings point to the potential influence of socioeconomic status on the development of problematic behaviors like internet addiction and gaming addiction. Socioeconomic status and technology use are additional external factors, which may impact sleep quality, and which have been reported as important risk factors for the experience of mental health problems^75–77^. While this has been demonstrated for gaming studies in developing countries^73,76^, the present study indicates there are also relationships between experiencing sleep disorder symptoms and gaming in Africa^1^. It is important to pay attention to the protective effect of being engaged or being married against problematic and addicted gaming. Our findings show that risks of insomnia, excessive daytime sleepiness, anxiety and depression decreased when a gamer is engaged or married. It is possible that the presence a partner reduces the time one can spend gaming and therefore, avoid problematic or addicted behaviors. The same observation is true for workers and student-workers who seem to have less problematic behaviour than students, according to our findings. The majority of studies related to gaming were made with students and showed that prevalence of problematic behaviour is high in this population^12,78^. None of these studies really evaluated the protective factor that being a student-worker or a worker may have on problematic gaming. Our findings raised the question about how occupation and employment may influence problematic behaviours, and more research is required to answer this question.

The effects of gaming on cognition, circadian rhythms as well as mood disorders are not well understood. Our findings pointed out the effects of gaming on four neuropsychiatric disorders including sleep disorders which have a lot of interactions with cognition and mood disorders(ref). The quantity, quality, and timing of sleep and wakefulness are regulated by both a homeostatic and a circadian process^79^. Deprivation of sleep has many negative consequences including cognitive impairment, metabolic dysregulation, and following extended sleep deprivation, eventually death^80,81^. In the same time, sleep disorders and circadian disruption are both associated to cognitive impairments and mood disorders^82^. Recent studies reported that gaming affects sleep and anxiety among adolescents and university students^9,20,83^. Knowing that both sleep and anxiety are directly associated with cognitive functions such as vigilance, attention and memory in the same populations^43,84,85^; it is reasonable to believe in an association between gaming and circadian rhythm. If a gamer plays during the night or in the dark of his/her room, circadian rhythm may be disturbed because of device backlighting. It was demonstrated that the lack of exposure to the daylight can induce apoptosis in monoaminergic systems in association with behavioural depressive phenotype^86^. All this evidence put together suggests a possible link between gaming and circadian disruption, and an interplay between depression and problematic gaming. More research is necessary to improve knowledge on these relations.

The languages used in the questionnaire (French and English) may be a limitation. Many countries where the research was performed have an additional language which citizens use on a daily basis. The questionnaire was available in French and English, but it may have been possible to increase the response rate if the questionnaire was available in other languages, such as Arabic (which is the common language in Tunisia and Morocco) and Kinyarwanda (which is the main language spoken in Rwanda in equal proportion of French, English and Swahili). The second limitation is the number of respondents who replied to the questionnaire. A total of 53,634 invitations were sent to potential participants and 12,680 forms were returned (response rate = 23.64%). This may be due to a lack of interest for the research, or because of the cultural habits where empirical and biomedical research are not well embedded in culture and inside the African healthcare system^87^. It can also be caused by the effects of individuals being fed up with being asked to complete surveys and questionnaires more frequently (e.g., questionnaire issuing for marketing, survey made for advertising purpose, questionnaires shared through social media like Facebook and WhatsApp, survey inside mobile games or AppStore), in addition to the perceived risk of a breach in confidentiality which may decrease people’s motivation to participate in research^88^.

This study points to the necessity for the global research community to pay more attention to low- and middle- income countries, in regard to the prevalence and incidence of sleep disorders and mood disorders, and research on internet gaming addiction. There is still a lot unknown in relation to diseases associated with gaming and the sociodemographic and environmental risk factors. Furthermore, associations with mental health disorders are missing specifically for low- and middle- income countries; and in particularly for African countries. It is also important to investigate their distribution in the general population because most studies reported gaming problems for students in colleges and universities; while those not studying may face similar problems. Men seem to be more affected by gaming, because the majority of gamers were males and the proportion of problematic gamers and addicted gamers were higher for men than women. The present research suggests that environmental factors such as socioeconomic status may affect the choice of device used for gaming, and so influence the development of problematic use of technologies or the development of an addiction to gaming. Similarly, more attention should be paid to the sleep of gamers. More research on gaming addiction needs to be performed in different geographical regions where little is known about internet gaming disorder.

## Data Availability

Data are available upon request made to the main author at faustin.armel.etindele.sosso@umontreal.ca.
